RETRACTED

# Clinical Effectiveness of Free Upper Arm Medial Flap in Repairing Skin and Soft Tissue Defects of the Dorsum of the Hand

**DOI:** 10.1155/2022/7144037

**Published:** 2022-06-26

**Authors:** Xuejun Yu, Wen Zheng, Wei An, Shengtao Xiang, Linglong Zhao

**Affiliations:** Department of Handsurgery, 521 Hospital of Norinco Group, Xi'an, Shaanxi, China

## Abstract

**Objective:**

To study the effectiveness of medial upper arm free flap in repairing skin and soft tissue (SST) defects of the dorsum of the hand.

**Methods:**

10 patients with SST defects on the dorsum of the hand who underwent free upper arm medial flap repair in our hospital from March 2017 to August 2018 were included in the study. Hand function, flap survival rate, wound healing, donor wound recovery, and the level of pain in the injured area were recorded before the operation, 1 month, and 6 months postoperatively.

**Results:**

The highest score in hand function was seen at the 6-month postoperative interval, followed by that at the 1-month postoperative interval. The lowest score in hand function was the preoperative score (*P* < 0.05). All flaps were still surviving 6 months postoperatively. Recovery of the function of the donor muscle, the elbow joint, as well as wound healing, all progressed well. 6 months postoperatively, 3 patients developed numbness and stiffness of the hand, but the symptoms were relieved following treatment. Compared to the preoperative scores, the visual analogue scale (VAS) scores at the injured site 1 month and 6 months postoperatively were significantly decreased, with the 6-month postoperative score being lower than the 1-month postoperative score (*P* < 0.05).

**Conclusion:**

The free upper arm medial flap is a good alternative for repairing skin and soft tissue defects of the dorsum of the hand with exposed phalanges, an approach that merits widespread promotion and clinical application.

## 1. Introduction

Skin and soft tissue (SST) defects of the opisthenar (i.e., the dorsum of the hand), common following traumatic hand injury, may be accompanied by an exposed or fractured phalanx, ruptured tendon, or considerably severe injury [1–3]. Generally, skin flaps of corresponding sizes should be isolated from other parts of the patient's body to repair the soft tissue at the back of the hand following trauma. At present, common donor sites for the skin flaps include the dorsum of the foot, the anterolateral thigh, and the lateral arm. However, the skin flaps are more bloated, and the survival rate of the skin flaps after repair is not impressive, which in turn poses a negative impact on both the recipient and the donor sites [4–6]. It has been reported that flaps from the medial aspect of the upper arm can be used to repair SST defects of the opisthenar, with desirable effectiveness [7]. This study aims to determine the effectiveness of free upper arm medial flaps at repairing SST defects of the opisthenar, by selecting patients with SST defects and exposed phalanges, and analyzing the survival rate of the flap and the recovery of donor-recipient function after repair.

RETRACTED

## 2. Data and Methods

### 2.1. General Data

10 patients with SST defects of the opisthenar with exposed phalanges admitted to our hospital from March 2017 to August 2018 were selected, with 7 of them being male, and 3 of them being female. All patients were aged between 24 and 50 years old, with an average age of 33.45 ± 5.49 years old. The duration from injury occurrence to hospital admission was 2.94 ± 0.88 hours. The causes of injury range from grinding wheel abrasion, to thermal crushes, mechanical injuries, and crushing injuries. 6 patients sustained injuries to the right hand, and 4 patients sustained injuries to the left hand. 7 patients had skin and soft tissue defects on the back of the fingers, while 3 patients had their defects behind the wrist. The average area of the defect 4.33 ± 0.61 cm^2^, and all defects were accompanied by phalangeal exposure, phalangeal fracture, and tendon exposure. 1 case had combined extensor tendon defects from the first to the fifth finger, 1 case had combined extensor tendon defects of the thumb, the index, and the middle fingers, 5 cases had combined extensor tendon defects from the second to the fifth finger, 2 cases had combined extensor tendon defects of the index, middle, and ring fingers, and lastly, 1 case had combined extensor tendon defects of the index and middle fingers. Refer to Table 1 for patient demographics.

### 2.2. Inclusion/Exclusion Criteria

#### 2.2.1. Inclusion Criteria

① Patients with SST defects of the opisthenar;
② Patients without other organic diseases, and with normal heart, lung, and kidney functions;
③ Patients aged at least 18 years;
④ Patients in whom this study is not contraindicated; it is worth stating that approval from the ethics committee and informed consent from all the patients involved in this study were duly obtained.

#### 2.2.2. Exclusion Criteria

① Patients with coagulation disorders or taking anticoagulants;
② Patients suffering from diabetes, hypertension, and other chronic diseases;
③ Patients that recently underwent major surgery;
④ Patients with damage to vital nerves or blood vessels;
⑤ Patients with a combination of fractures and other complex injuries to the hand.

### 2.3. Methods

Patients with mildly contaminated injuries can be treated directly with free upper arm medial skin flap repair, following cleaning of the wound. Patients with moderate to severely contaminated injuries should first be treated with surgical debridement, dressing change, and anti-inflammatory agents. When the wound is dry, free of purulent secretions, and the general condition of the patient is good, free upper arm medial skin flap repair is then performed on a selective basis.

RETRACTED

The patient is placed in a supine position, with the upper arm tied with a tourniquet. A local anesthetic is given, and the wound is routinely disinfected. Afterwards, the fractured end of the phalanx is reset and fixed, and the injured tendon is sutured using an 8-gauge suture [8–10]. The size of the wound at the back of the hand is then measured. A Doppler ultrasound blood flow detector (GE Medical Systems Kretztechnik GmbH & Co. OHG; Batch number: 2003 No. 3230478) is used to locate the flap on the medial aspect of the upper arm, using the line joining the tip of the axilla and the medial epicondyle of the humerus as the center line. The size of the flap is estimated using the formula:

(1) $$\begin{array}{c} \text{Flap size}=\text{area of the defect on the opisthenar}\times 110\%. \end{array}$$

When cutting the flap, it is essential that the ulnar nerve and blood vessels are protected. Next, the donor wound is sutured. The upper arm flap is placed at the SST defect of the opisthenar, and the edge is fixed. Then, the vascular pedicle in the flap is anastomosed to the corresponding blood vessels of the hand, with the nerve of the flap being anastomosed to the corresponding nerve of the opisthenar. Lastly, after performing the above mentioned procedures, the final suture is performed (Figure 1).

### 2.4. Observation Indicators

Hand function, flap survival rate, wound healing, donor wound recovery, and the level of pain at the injured site were recorded before the operation, 1 month, and 6 months after the operation.

1. Assessment of upper limb function [11]: this was based on such factors as range of motion of the joints, muscle strength, sensation, appearance, residual symptoms, and working conditions. A score of 80–100 is considered excellent, 60–79 is considered good, 40–59 is considered poor, and that of <39 is considered poor.
2. Survival of the skin flap was determined by the activity of the skin flap, and blood flow detection was determined using Doppler ultrasound.
3. Degree of pain: the visual analogue scale (VAS) was used to evaluate the degree of pain at the injured site, with a score of 0 corresponding to no pain, and that of 10 corresponding to severe pain. The higher the VAS score, the more intense the pain, and vice-versa.

RETRACTED

### 2.5. Statistical Analysis

SPSS20.0 was used as the data processing software, and GraphPad Prism 7 (San Diego, USA) was used as well. The measuring data was expressed as ($\bar{x}\pm s$), and the *t*-test was carried out. The counting data was expressed as (*n* (%)), and the *X*^2^ test was carried out.

## 3. Results

### 3.1. Comparison of Hand Function Preoperatively, 1 Month, and 6 Months Postoperatively

The preoperative trauma of patients is shown in Figure 2. The hand function scores of all patients were assessed preoperatively, 1 month, and 6 months postoperatively, and then compared. The highest score in hand function was seen at the 6 month postoperative interval, followed by that at the 1 month postoperative interval. The lowest score in hand function was the preoperative score, with significant statistical significance (*P* < 0.05). These findings are illustrated in Figure 3.

### 3.2. Recovery 1 Month and 6 Months Postoperatively

All patients were observed for flap survival rate 1 month and 6 months postoperatively. The results showed that all the flaps were still surviving 1 month and 6 months postoperatively, and that the patients could freely move their hands. 6 months postoperatively, 3 patients developed numbness and stiffness of the hand, but the symptoms were relieved following administration of mecobalamin tablets, and completely disappeared after a week of treatment. Also, the scar at the donor site was significantly reduced 6 months postoperatively. This, coupled with the fact that the position of the scar is relatively hidden (on the medial aspect of the upper arm), greatly minimizes the impact of the scar on the patient's daily life. See Figures 4–6 for illustration.

### 3.3. Pain at the Injured Site

Pain at the injured site was assessed before surgery, as well as 1 month and 6 months after surgery. Compared to the preoperative scores, the visual analogue scale (VAS) scores at the injured site at the 1-month and 6-month postoperative intervals were significantly decreased, with the 6-month postoperative score being lower than the 1-month postoperative score (*P* < 0.05). See Figure 7 for illustration.

## 4. Discussion

SST defects of the dorsum of the hand need to be repaired using flaps isolated from other parts of the patient's body [12–14]. The traditional approach involves changing the dressing after thorough debridement, or applying a negative pressure drainage device to cover the wound surface, and then, following growth of granulation tissue on the wound surface, free skin grafting is performed. This method requires multiple operations, a longer period of treatment, and a relatively long wound exposure time, which is likely to cause secondary infection and deep tissue necrosis. Additionally, postoperative wounds are prone to scar contracture, and recovery of hand function is usually poor [15, 16]. There are abundant vascular perforations in the skin of the medial aspect of the upper arm, and both the skin and tissue are similar to those at the dorsum of the hand. It has been reported that using a flap isolated from the medial aspect of the upper arm to repair skin and soft tissue defects of the dorsum of the hand is associated with good recovery, and a very low incidence of adverse reactions [17, 18]. Flaps isolated from the medial aspect of the upper arm site have a good texture and a beautiful appearance, factors which combine to make the site a good candidate for the isolation of flaps to be used in the repair of skin and soft tissue defects of the dorsum of the hand. In this study, flaps from the medial aspect of the upper arm flap were used for repair of skin and soft tissue defects of the dorsum of the hand. Our study subjects were drawn from patients with SST defects of the opisthenar with fractured or exposed phalanges, and exposed or ruptured tendons. A free flap isolated from the medial aspect of the upper arm was used to repair the SST defects of the opisthenar. The hand function of the patients was assessed before the operation, 1 month, and 6 months postoperatively, and then compared. Also, the recovery of the wounds at the donor and recipient sites was assessed 1 month and 6 months postoperatively.

RETRACTED

In this study, all the flaps were still surviving 1 month and 6 months postoperatively. The patients had the highest score in hand function at the 6 month postoperative interval, followed by that at the 1 month postoperative interval. The lowest score in hand function was seen preoperatively. With extended recovery times, higher scores in hand function, and better hand function recovery were seen in all the patients. 6 months postoperatively, 3 patients developed numbness and stiffness of the hands, but the symptoms were relieved following treatment with muscle relaxants, disappearing completely after one week of treatment.

Similar to the findings obtained by the research conducted by Wang et al. [19], the skin in the medial aspect of the upper arm is considered thin, soft and elastic enough to allow it to be used clinically for the repair of small and medium sized skin and soft tissue defects of the dorsum of the hand. This study shows that using flaps isolated from the medial aspect of the upper hand is an effective way of repairing skin and soft tissue defects of the dorsum of the hand, and is associated with good recovery of hand function, as well as good wound healing at the donor and recipient sites. The study also shows that this approach is associated with a significantly lower degree of postoperative pain, which, to a decent extent, enhances the confidence of the patient and the reliability of the study.

RETRACTED

## 5. Conclusion

In conclusion, flaps isolated from the medial aspect of the upper arm are a good option for repairing skin and soft tissue defects of the dorsum of the hand. This approach is one that merits more widespread clinical application.

## Figures and Tables

**Figure 1:** Surgical procedure.

**Figure 2:** Preoperative trauma.

**Figure 3:** Comparison of hand function preoperatively, 1 month, and 6 months postoperatively. The figure shows the preoperative, 1 month, and 6 month postoperative scores in hand function (from left to right). Hand function score was 36.54 ± 5.99 preoperatively, 59.82 ± 8.73 1 month postoperatively, and 81.06 ± 10.22 6 months postoperatively. ^∗^Compared with preoperative, *P* < 0.001; ^#^Compared with 1 month postoperatively, *P* < 0.001.

**Figure 4:** Recovery at the recipient site in the immediate postoperative period.

**Figure 5:** Recovery at the donor site 1 month postoperatively.

**Figure 6:** Recovery at the recipient site 6 month postoperatively.

**Figure 7:** Pain levels at the injured site before surgery, 1 month, and 6 months after surgery, expressed as VAS score (from left to right). VAS score was 7.64 ± 0.86 preoperatively, 5.67 ± 1.21 1 month postoperatively, and 2.12 ± 0.68 6 months postoperatively.

**Table 1:** Patient demographics.

	Male (*n* = 7)	Female (*n* = 3)	Total (*n* = 10)
Age (years)	35.49 ± 3.23	36.37 ± 3.25	36.42 ± 2.98
Area of defect (cm^2^)	4.25 ± 0.58	4.34 ± 0.59	4.33 ± 0.61
Interval from injury to hospital admission (hrs)	2.87 ± 0.76	2.97 ± 0.75	2.94 ± 0.88

## Data Availability

The datasets used and analyzed during the current study are available from the corresponding author on reasonable request.

## Abbreviations

SST: Skin and soft tissue.
